# An Integrated Approach Fusing CEEMD Energy Entropy and Sparrow Search Algorithm-Based PNN for Fault Diagnosis of Rolling Bearings

**DOI:** 10.1155/2022/4835157

**Published:** 2022-07-22

**Authors:** Yue Xiao, Zhiqing Zeng, Ziyang Deng, Chao Lin, Zuquan Xie

**Affiliations:** School of Mechanical Engineering, Nanchang Institute of Technology, Nanchang, Jiangxi 330099, China

## Abstract

This paper solves the problem of difficulty in achieving satisfactory results with traditional methods of bearing fault diagnosis, which can effectively extract the fault information and improve the fault diagnosis accuracy. This paper proposes a novel artiﬁcial intelligence fault diagnosis method by integrating complementary ensemble empirical mode decomposition (CEEMD), energy entropy (EE), and probabilistic neural network (PNN) optimized by a sparrow search algorithm (SSA). The vibration signal of rolling bear was firstly decomposed by CEEMD into a set of intrinsic mode functions (IMFs) at different time scales. Then, the correlation coefficient was used as a selection criterion to determine the effective IMFs, and the signal features were extracted by EE as the input of the diagnosis model to suppress the influence of the redundant information and maximize the retention of the original signal features. Afterwards, SSA was used to optimize the smoothing factor parameter of PNN to reduce the influence of human factors on the neural network and improve the performance of the fault diagnosis model. Finally, the proposed CEEMD-EE-SSA-PNN method was veriﬁed and evaluated by experiments. The experimental results indicate that the presented method can accurately identify different fault states of rolling bearings and achieve better classification performance of fault states compared with other methods.

## 1. Introduction

Rolling bearings often work under complex operating conditions such as heavy load, impact, and variable speed. The faults of rolling bearings may seriously affect the normal operation of mechanical equipment and even cause safety accidents. Therefore, the condition detection and fault diagnosis of rolling bearings are of great significance to ensure the safe operation of mechanical equipment [1]. Feature extraction and classiﬁcation identiﬁcation are the most important parts in the bearing fault diagnosis process.

Effectively extracting the features of the rolling bearings is the key to recognize different fault states in the fault diagnosis [2]. However, the early fault signal of bearing is weak and easy to be corrupted by noise, which will make the fault feature extraction difficult. In addition, the vibration signal has the characteristics of nonlinearity and nonstationary due to the vibration coupling of mechanical system and the influence of complex environment, which will make it hard to extract fault features only from the perspective of time domain, frequency domain, or time-frequency domain [3]. Presently, some signal analysis methods, such as wavelet transform (WT), empirical modal decomposition (EMD), ensemble empirical modal decomposition (EEMD), complementary ensemble empirical mode decomposition (CEEMD) as well as variational mode decomposition (VMD), have been applied to extract signal features. The WT method has good time-frequency localization characteristics but lacks self-adaptation due to difficulties in determining wavelet basis and decomposition levels [4]. The EMD method proposed by Huang et al. [5] adaptively decomposes a signal into the sum of several intrinsic modal functions (IMFs), which has good decomposition performance and can stabilize the nonstationary data. This method is considered as a significant breakthrough of traditional time-frequency analysis methods and has been frequently applied in the field of mechanical fault diagnosis. However, it suffers from the drawbacks of mode mixing and endpoint effects [6, 7]. The EEMD method is proposed to reduce the mode mixing by adding Gaussian white noise with different values to the original signal, which can make the extreme point distribution in the original signal change and reliably eliminate the phenomenon of modal aliasing. For avoiding interference from the added Gaussian white noise, the mean value of the decomposed results is solved based on the zero-mean characteristics of the Gaussian white noise. With the increase of the number of operations to calculate the mean value, the decomposition results will be less affected by the added Gaussian white noise. However, EEMD clearly has the disadvantages of excessive iterative loss time and low decomposition accuracy [8, 9]. Yeh et al. [10] proposed the CEEMD method to further suppress the adverse effects of Gaussian white noise on the reconstruction of the original signal. Unlike the EEMD method, which only adds Gaussian white noise to the original signal once during the operation of averaging, CEEMD introduces the corresponding opposite value on the basis of adding Gaussian white noise, and realizes the operation of adding positive and negative Gaussian white noise to the signal, respectively, to perform double averaging. Therefore, CEEMD can more thoroughly eliminate the reconstruction error caused by the addition of Gaussian white noise [11, 12]. The VMD algorithm is a nonrecursive signal decomposition method proposed by Dragomiretskiy and Zosso [13], which uses an iterative search for the optimal solution of the variational model to determine the frequency center and bandwidth of each decomposition part. It can transform the constrained variational problem into a nonconstrained one by introducing a quadratic penalty factor and Lagrangian multiplication operator, and has a complete mathematical basis and solution method. Huang et al. [14] proposed a modiﬁed scale-space VMD to improve the adaptability of variational mode decomposition and computational efﬁciency. Lv et al. [15] studied a support vector machine algorithm based on VMD and refined the composite multiscale dispersion entropy to realize the rapid and effective identification of bearing fault types. However, the VMD method has the problem of selecting the proper decomposition parameters including the mode number and bandwidth control parameter. If the two parameters are optimized independently and the interaction between them is neglected, it would cause a trap in local optimization. The intelligence optimization algorithms are prevalent options for the optimizing of VMD decomposition parameters. However, there is no unified standard for the construction of objective function for the VMD parameter optimization, such as kurtosis, entropy, and correlation coefﬁcient, which directly inﬂuences the performance of decomposition. To achieve the optimal selection of the two parameters in VMD, Zhang et al. [16] propose a parameter-adaptive VMD by using the grasshopper optimization algorithm to improve the performance of VMD, in which the maximum weighted kurtosis index was used as optimization objective. Gai et al [17] utilized the hybrid grey wolf optimizer algorithm to search for the optimal parameter combinations in VMD for the early fault diagnosis of rolling bearing. Recently, Ni et al. [18] proposed a fault information-guided VMD (FIVMD) method for extracting the weak bearing repetitive transient under complicated operating conditions, which used the generalized Gaussian cyclostationary (GGCS) model and the generalized Gaussian stationary (GGS) model to determine the mode number, and employed the ratio of fault characteristic amplitude (RFCA) to identify the optimal bandwidth control parameter.

After feature extraction, classiﬁcation identiﬁcation is another critical step to fault diagnosis by using an intelligent pattern classifier. In essence, fault diagnosis can be regarded as a process of fault pattern recognition. Early classiﬁcation identiﬁcation mainly depends on manual experience, which has great limitations in terms of real-time and accuracy of fault diagnosis. Current development of mechanical equipment is in the direction of high speed, high precision, and high efficiency; the field of mechanical health detection has entered the era of big data, artificial intelligence, and machine learning technologies which have been widely used in intelligent fault diagnosis of mechanical equipment. A series of artificial intelligence methods such as support vector machines (SVM) [19, 20], k-nearest neighbor (KNN) [21], convolutional neural network (CNN) [22, 23], artificial neural network (ANN) [24], recurrent neural network (RNN) [25], gated recurrent unit (GRG) [26], etc., have been used in the field of fault diagnosis. The application of the artificial intelligence methods can make progressively the fault diagnosis of rolling bearings more efficient and effective. However, there still reminds some challenges while developing the artificial intelligence and machine learning methods including local minimum and over-fitting.

Probabilistic neural network (PNN) [27] is an intelligent algorithm based on Bayesian decision theory and Parzen window probability density function and is developed on the basis of radial basis function neural network. Compared with other artificial intelligence methods, the computational process of PNN is relatively simple, and it has a fast convergence rate in running computation, with results always converging to the Bayesian optimal solution. Moreover, PNN has ultra-high stability and strong fault tolerance for individual abnormal data, especially in the field of fault diagnosis. For newly added or deleted sample data, it does not need retraining, while maintaining high classification accuracy and can also meet the requirements of modification at any time in sample training. Liu et al. [28] proposed a fault diagnosis algorithm which combines CEEMD and energy moment calculation with PNN algorithm to improve the performance on the feature extraction from bearing signals and the accuracy of the fault diagnosis. Zhao et al. [29] combined fast iterative filter decomposition with PNN to decompose the bearing signal into several eigen modal functions and extract the EE values as the feature vector, which can rapidly and accurately identify the faults at different positions of the bearing.

As the only input parameter for PNN, the choice of smoothing factor has a great inﬂuence on the final identification performance of the network model. However, the smoothing factor in traditional PNN depends on empirical values and lacks self-adaptability [30]. Therefore, it is essential to optimize the smoothing factor of PNN to improve the classiﬁcation accuracy and calculation speed. Although many traditional optimization algorithms have carried out relevant research, some deterministic methods, such as the Lagrange, conjugate gradient, and simplex method, cannot provide a fitting solution with highly nonlinear search domains in PNN and are easy to get trapped in local optimal solutions [31]. Exploring the most suitable smoothing factor of PNN by using such deterministic methods is not always possible or feasible. In recent years, the swarm intelligence algorithm has been applied because of its simple structure and high solving efficiency in the fields of machine learning, process control, and pattern recognition. As a meta-heuristic optimization algorithm, the swarm intelligence optimization algorithm imitates the behavior of biological populations or natural phenomena in nature, which has intelligent characteristics such as self-adaptation, self-learning, and self-organization, and is convenient for large-scale parallel computing. There have been many different swarm intelligence optimizations available in the existing literature. Among them, genetic algorithm (GA) and particle swarm optimization (PSO) algorithm are the most representative methods and have been successfully applied in many engineering problems [32]. Currently, more and more new swarm intelligence algorithms are proposed, such as bat algorithm (BA) [33], monarch butterfly optimization (MBO) [34], slime mould algorithm (SMA) [35], moth search algorithm (MSA) [36], hunger games search (HGS) [37], Runge Kutta method (RUN) [38], colony predation algorithm (CPA) [39], weIghted meaN oF vectOrs (INFO) [40], and Harris hawks optimization (HHO) [41].

Sparrow search algorithm (SSA) [42] is a new swarm intelligence optimization algorithm based on the foraging and anti-predation behaviors of sparrows proposed by Xue et al. In detail, SSA has the advantages of fast convergence, high search accuracy, and good stability, which can help the population to find the optimal solution more quickly. Li et al. [43] provided a review of relevant studies on six more typical swarm intelligence algorithms proposed since 2010, including BA, grey wolf optimization (GWO), dragonfly algorithm (DA), whale optimization algorithm (WOA), grasshopper optimization algorithm (GOA), and SSA, and further compared the experimental performance of these algorithms by using 22 standard CEC test functions in terms of the convergence speed, accuracy, stability, and robustness. From the comprehensive comparison of the experimental results, the performance of the SSA proposed in 2020 is far superior to the other five optimization algorithms, and it has great potential. Therefore, this paper employs SSA to optimize the parameters of PNN.

In view of the drawbacks of the abovementioned feature extraction methods and the limitations of classiﬁcation identiﬁcation, in this paper, a method combining CEEMD and PNN is proposed to identify the fault type of rolling bearings. The vibration signal is decomposed into a series of IMFs by CEEMD, and the energy entropy (EE) value of the first few IMF components with high correlation are estimated. The difference of the EE values under different working conditions can effectively reflect the characteristics of fault type. Extract the EE values to form a feature vector to input into PNN, which was chosen as the basis for the fault diagnosis classiﬁer. Since the classiﬁcation performance of PNN is easily affected by the smoothing factor, the PNN model optimized by sparrow search algorithm is used to train and identify the different fault states of rolling bearings. The effectiveness of the proposed method is analyzed through the measured rolling bearing test. Experimental results show that the fault diagnosis performance of the proposed method is better than that of other similar fault diagnosis methods of rolling bearings.

The remainder of this paper is organized as follows: Section 2 introduces the related theories of the proposed method. The overall procedure of the proposed fault diagnosis model is presented in Section 3.  Section 4 presents the simulation experiment to verify the proposed method in decomposition performance. In Section 5, the proposed fault diagnosis model based on CEEMD, EE, and SSA-optimized PNN is validated in comparison experiments.  Section 6 draws the conclusions of this work.

## 2. Theoretical Background

### 2.1. Complementary Ensemble Empirical Mode Decomposition

This work selects CEEMD to process the original vibration signal, which is the improvement of EMD and CEEMD. The traditional EMD is able to adaptively decompose a nonstationary time-series signal into a series of relatively stable intrinsic mode components (IMFs) as well as a standard residual in which each IMF reflects the dynamic characteristics of the original signal. However, some nonlinear signals with abnormal interference can produce modal aliasing, resulting in the appearance of different time-scale characteristics simultaneously in the same modal component. EEMD adds Gaussian white noise to the original signal and takes advantage of the uniform feature of Gaussian white noise spectrum to make the signals of different time scales automatically distributed to a suitable reference scale, which can effectively suppress modal aliasing. However, the implementation of repeated decomposition of the signal several times and averaging by EEMD do not eliminate the effect of the added Gaussian white noise on the decomposition results, and the operation efficiency is low.

The CEEMD algorithm can solve the interference of Gaussian white noise and the problem of generating error in signal reconstruction. The empirical modal and empirical modal decomposition of the two groups of signals, respectively, by adding a pair of Gaussian white noise with the same phase but opposite amplitude to the original signal can significantly reduce the reconstruction error since the added Gaussian white noise is neutralized. The CEEMD method not only effectively solves the problem of mode mixing caused by EMD but also overcomes the defect of the incompleteness of signal reconstruction by EEMD [44]. The concrete steps of CEEMD are as follows:

(1) Set the total aggregation time *M* and the root mean square (RMS) amplitude of added Gaussian white noise *a,* and *i* = 1.
(2) Add a pair of Gaussian white noise with the same phase but opposite amplitude to the original signal to obtain two new sets of signals
  (1) $$\begin{array}{c} \left\{\begin{array}{c} p_{i}^{+}\left(t\right)=x\left(t\right)+n_{i}\left(t\right),\\ p_{i}^{-}\left(t\right)=x\left(t\right)-n_{i}\left(t\right), \end{array}\right. \end{array}$$
where *x*(*t*) is the original signal, *n*_*i*_(*t*) is the added Gaussian white noise for *i*th time, *p*_*i*_^+^(*t*) and *p*_*i*_^−^(*t*) represent the signal after adding positive and negative Gaussian white noise for the *i*th time, respectively.
(3) Decompose *p*_*i*_^+^(*t*) and *p*_*i*_^−^(*t*), respectively, by EMD to obtain two sets of IMF components, and the number of components in each group is *K*, then
  (2) $$\begin{array}{c} \left\{\begin{array}{c} p_{i}^{+}\left(t\right)=\sum_{j=1}^{K}c_{i,j}^{+}\left(t\right)+r_{i}^{+}\left(t\right),\\ p_{i}^{-}\left(t\right)=\sum_{j=1}^{K}c_{i,j}^{-}\left(t\right)+r_{i}^{-}\left(t\right), \end{array}\right. \end{array}$$
where *c*_*i*,*j*_^+^(*t*) and *c*_*i*,*j*_^−^(*t*) are the *j*th IMF component decomposed after adding Gaussian white noise for the *i*th time, *K* is the number of IMF components, *r*_*i*_^+^(*t*), and *r*_*i*_^−^(*t*) are the residuals after decomposition.
(4) *i* = *i* + 1, repeat steps (2) and (3) until the condition *i* = *M* is satisﬁed. Noted that the magnitude of Gaussian white noise is different for each addition with the different *i.*
(5) Take the average value of all IMF components after *M* times of decomposition as the final IMF components
  (3) $$\begin{array}{c} c_{j}\left(t\right)=\frac{1}{2M}\sum_{i=1}^{M}\left[c_{i,j}^{+}\left(t\right)+c_{i,j}^{+}\left(t\right)\right], \end{array}$$
where *c*_*j*_(*t*) is the *j*th IMF component obtained by the CEEMD, *j*=1,2, ⋯, *K*.

The diﬀerence between the original signal and the sum of all IMF components obtained by CEEMD can evaluate the effect of the added white noise on the decomposition results as follows:

(4) $$\begin{array}{c} \varepsilon =\frac{a}{\sqrt{M}}, \end{array}$$

where *ε* is the ﬁnal standard deviation of the reconstruction error.

Reducing the value of *a* contributes to improve the decomposition accuracy, and the value of *a* is usually taken as 0.1–0.3 times of the standard deviation of the original signal. When *a* is small to a certain degree, it is not enough to cause the local extreme points of the signal to change, and failing to alter the local time span of the original signal makes it difficult to achieve the goal of utilizing as many scales as possible to analyze the signal. On the other hand, increasing *M* also decreases the reconstruction error but greatly increases the computation time. When *M* is 100–300, the error caused by the residual white noise can be small enough in general, and increasing the execution time does not significantly improve the decomposition accuracy.

### 2.2. Correlation Coefficient Criterion

The IMFs decomposed by CEEMD are arranged from high frequency to low frequency; however, the IMFs with high frequency may contain random noise and the IMFs with low frequency may contain trend terms, spurious components, and residual components due to interpolation error and boundary effect. Only a part of IMFs can characterize the essential nature of the original signal, while the rest are some false mode components caused by noise. Therefore, the invalid IMF components need to be removed to maximize the retention of original signal features.

The correlation coefficient was applied as the criterion to select the effective IMF components, which is an important parameter to evaluate the correlation degree between the original vibration signal and each decomposed IMF component. If the correlation coefficient of the component is large, it indicates that the correlation between the component and the original signal is strong, in which the bearing operating state features contained are abundant. On the contrary, it shows that the bearing operation state characteristics contained in this component are less, and even there may be false components, which will disturb the fault diagnosis. By calculating the correlation coefficient between each IMF component and the original signal, the IMFs with relatively large correlation coefficient can be selected to represent the effective information in the original signal. The correlation coefficient can be deﬁned as follows:

(5) $$\begin{array}{c} C_{r}\left(j\right)=\frac{\sum_{i=1}^{N_{d}}\left(c_{j,i}-{\bar{c}}_{j}\right)\left(x_{i}-\bar{x}\right)}{\sqrt{\sum_{i=1}^{N_{d}}{\left(c_{j,i}-{\bar{c}}_{j}\right)}^{2}}\sqrt{\sum_{i=1}^{N_{d}}{\left(x_{i}-\bar{x}\right)}^{2}}}, \end{array}$$

where *C*_*r*_(*j*) is the correlation coefficient between the *j*th IMF component *c*_*j*_(*t*) and the original signal *x*(*t*), *N*_*d*_ is the number of data points, *x*_*i*_ is the *i*th data point of the original signal *x*(*t*), *c*_*j*,*i*_ is the *i*th data point of the *j*th IMF component *c*_*j*_(*t*), ${\bar{c}}_{j}$ and $\bar{x}$ are the average values of the corresponding signal data points, respectively.

In this way, the original signal can be reconstructed using IMF components filtered by the correlation coefficient principle, resulting in effective suppression of noise to ensure the accuracy of subsequent feature extraction and fault diagnosis.

### 2.3. Energy Entropy

Entropy is a powerful tool to analyze the dynamic changes of signals, which can represent the disorder degree of a complicated signal. The purpose of extracting feature information can be achieved by using the characteristic that entropy can effectively detect the complexity of the vibration signal of the bearing in case of fault. When the bearings operate in different states, there is a great difference in the energy of vibration signals, and the distribution of the energy in different frequency bands will change. Therefore, the different signal energy distribution of the bearing under different working conditions can be used as the basis for identifying the fault type. As an information entropy feature extraction method, energy entropy can characterize the signal change from the perspective of energy change. Here, energy entropy is introduced to judge different fault states of rolling bearings.

Given *h* effective IMF components selected by the correlation coefficient criterion, the energy value of each IMF component can be expressed as

(6) $$\begin{array}{c} E_{j}=\int_{-\infty }^{+\infty }{\left|c_{j}\left(t\right)\right|}^{2}\text{d}t,j=1,2,\cdots ,h, \end{array}$$

where *E*_*j*_ is the energy value of the *j*th IMF component.

The total energy of *h* effective IMF components can be calculated as

(7) $$\begin{array}{c} E=\sum_{j=1}^{h}E_{j}. \end{array}$$

The proportion of the energy of each IMF component to the total energy is taken as its probability value as

(8) $$\begin{array}{c} P_{j}=\frac{E_{j}}{E}, \end{array}$$

where *P*_*j*_ is the proportion of the energy of the *j*th IMF component to the total energy.

Then, the EE values of each IMF component can be expressed as:

(9) $$\begin{array}{c} H_{j}=-\sum_{j=1}^{h}P_{j}\ln P_{j}, \end{array}$$

where *H*_*j*_ is the EE value of the *j*th IMF component.

### 2.4. Probabilistic Neural Network

Probabilistic neural network (PNN) is a radial basis network based on the theory of Bayesian decision, and Parzen window function, which can solve nonlinear problems with a linear learning algorithm and has the advantages of simple learning process, fast training speed, more accurate classiﬁcation, good fault tolerance, etc. The PNN structure is composed of four layers: input layer, pattern layer, summation layer, and output layer, as shown in Figure 1.

The function of the input layer is to receive the input feature vector *x*=[*x*_1_, *x*_2_, ⋯,*x*_*h*_]^*T*^ from the training set and directly transfer these values to the pattern layer without any operation, in which the dimension of the input vector is equal to the number of neurons in the input layer.

The pattern layer is connected to the input layer by connecting weights, and the number of neurons in the pattern layer is equal to the product of the training types and the number of samples, in which the Gaussian function of each sample, and the output function of the pattern layer is expressed as:

(10) $$\begin{array}{c} \phi_{ik}\left(x\right)=\frac{1}{{\left(2\pi \right)}^{h/2}\sigma^{h}}\exp\left[-\frac{{\left(x-x_{ik}\right)}^{T}\left(x-x_{ik}\right)}{2\sigma^{2}}\right], \end{array}$$

where *i*=1,2, ⋯, *b*, *k*=1,2, ⋯, *m*_*i*_, *b* is the number of all types of training samples, *m*_*i*_ is the number of *i*th type of training samples, *h* is the dimension of the testing sample vector *x* and the training sample vector *x*_*ik*_, *σ* is the smoothing factor, and *x*_*ik*_ is the *k*th center value of the *i*th type of training sample.

The summation layer averages the output weights of the neurons belonging to the same type of pattern layer and the result is as follows:

(11) $$\begin{array}{c} g_{i}\left(x\right)=\frac{1}{m_{i}}\sum_{k=1}^{m_{i}}\phi_{ik}\left(x\right), \end{array}$$

where *g*_*i*_(*x*) is the output of *i*th type of training samples in the summation layer.

The number of neurons in the summation layer is the same as the total number of pattern layer, and the neurons in this layer are only connected with the corresponding neurons in the pattern layer and will not be connected with other neurons.

The output layer is composed of competing neurons with the same number of neurons as the summation layer, in which each neuron corresponds to a kind of pattern, respectively. Its function is to receive the output generated by the summation layer and set the type corresponding to the highest probability in the network summation layer as the output result. The result is as follows:

(12) $$\begin{array}{c} y\left(x\right)=\underset{i=1,2,\cdots ,b}{\arg\max}\left\{g_{i}\left(x\right)\right\}. \end{array}$$

When the data and types of the training samples are determined, the structure of the probabilistic neural network and the number of neurons in each layer are fixed and the performance of the network model depends on the choice of smoothing factor *σ*. Since the smoothing factor is related to the correlation degree between the layers of the training sample, an optimization algorithm needs to be employed to select an appropriate smoothing factor.

### 2.5. Sparrow Search Algorithm

Sparrow search algorithm (SSA) is a novel intelligent optimization algorithm with fast convergence speed and strong optimization ability, which is proposed according to the behavior of sparrows foraging and escaping from predators. SSA takes into account all possible factors of population behavior, so that the algorithm can quickly converge to the optimal value with good global optimization ability and stability. The performance of SSA had been discussed in great detail by previous research work [42, 43], and the experimental studies have shown that SSA has strong competitiveness with good convergence speed and exploitation capability for the optimization of the unimodal test functions, multimodal test functions, and fixed-dimension test functions. Moreover, SSA has a good search ability to explore the potential region of the global optimum, and the local optimum can be avoided effectively. Overall, the SSA employed in this paper has the following advantages: (1) it is promising for real complex and challenging optimization problems with constrained and unknown search domains; (2) it is easy to implement, and has a strong ability to adapt to various types of optimization problems; (3) it has a good ability of global exploration and local exploitation; and (4) it has strong scalability, stability, and robustness.

The search process can be abstracted as a discoverer-follower-scouter model, and their identities constitute a dynamic balance in the sparrow population. The discoverer is responsible for guiding the population to forage, and the follower follows the discoverers to obtain food. Meanwhile, a certain proportion of individuals in the population are selected as scouters for detection and early warning, which keep alert to environmental threats and warn the sparrow population to move to closer to safe areas [45].

In the SSA model, the discoverers with good fitness evaluation are able to find the food area and obtain food first during the search process, and the discoverers have a larger foraging search range than the followers since they are responsible for providing the feeding direction for the sparrow population.

Assuming the number of sparrows is *R* and the dimensionality of the optimization variables is *D*, *X*_*r*_=[*X*_*r*,1_, ⋯, *X*_*r*,*d*_, ⋯, *X*_*r*,*D*_] is the position of the *r*th sparrow, *X*_*r*,*d*_ is the position of the *r*th sparrow in the *d*th dimension,*r*=1,2, ⋯, *R*. The position of the discoverer is updated during the iterative process as follows:

(13) $$\begin{array}{c} X_{r,d}^{t+1}=\left\{\begin{array}{cc} X_{r,d}^{t}\cdot \;\exp\left(-\frac{r}{\lambda \cdot t_{\max}}\right), & \text{if }V_{W}<V_{\text{ST}},\\ X_{r,d}^{t}+Q\cdot L, & \text{if }V_{W}\geq V_{\text{ST}}, \end{array}\right. \end{array}$$

where *t* is the current number of iterations, *d*=1,2, ⋯, *D*, *t*_max_ is the maximum number of iterations, *X*_*r*,*d*_^*t*^ is the current position of the *r*th sparrow in the *d*th dimension at iteration *t*, *λ* ∈ (0,1] is a random number, *V_W_* is the early warning value, *V*_ST_ is the safety threshold, and *V*_*W*_ ∈ [0,1], *V*_ST_ ∈ [0.5, 1]. *Q* is a random number with a normal distribution. *L* is a 1 × *D* matrix in which each element is 1. When *V*_*W*_ < *V*_ST_, the discoverer can perform an extensive foraging search, and there are no predators around foraging at this time. When *V*_*W*_ ≥ *V*_ST_, this indicates that there have been sparrows finding predators and alerting other sparrows in the population, the discoverer will lead other sparrows quickly to other safe areas for foraging.

The worse the foraging position of the followers in the group, the lower the corresponding energy will be. The followers can always find discoverers who provide rich resources during foraging, facilitating better food for them. To increase the chances of getting food, the followers will continuously monitor the discoverers and rob food resources. The position of the follower is updated as follows:

(14) $$\begin{array}{c} X_{r,d}^{t+1}=\left\{\begin{array}{cc} Q\cdot \;\exp\left(\frac{X_{W}^{t}-X_{r,d}^{t}}{r^{2}}\right), & \text{if }r>\frac{R}{2},\\ X_{p}^{t+1}+\left|X_{r,d}^{t}-X_{p}^{t+1}\right|\cdot A^{+}L, & \text{if }r\leq \frac{R}{2}, \end{array}\right. \end{array}$$

where *X*_*p*_ is the optimal position currently occupied by the discoverer, and *X*_*W*_ is the current global worst location. *A* is a 1 × *D* matrix in which each element is randomly assigned 1 or −1, and *A*^+^=*A*^*T*^(*AA*^*T*^)^−1^. When *r* > *R*/2, this indicates that the *r*th follower in the population does not get food and needs to ﬂy elsewhere to get more energy. When *r* ≤ *R*/2, this indicates that the *r*th follower will randomly seek a location for foraging near the current optimum.

When attacked by outsiders, the individual sparrows on the edge of searching and foraging will continuously adjust their position and move closer toward the inner safety area, and the individual sparrows in the inner safety area will try to get closer to their companions to increase their safety. The process of individual sparrows updating the location is as follows:

(15) $$\begin{array}{c} X_{r,d}^{t+1}=\left\{\begin{array}{cc} X_{B}^{t}+\beta \cdot \left|X_{r,d}^{t}-X_{B}^{t}\right|, & \text{if }f_{r}>f_{B},\\ X_{r,d}^{t}+u\cdot \left(\frac{\left|X_{r,d}^{t}-X_{W}^{t}\right|}{\left(f_{r}-f_{W}\right)+\varepsilon }\right), & \text{if }f_{r}=f_{B}, \end{array}\right. \end{array}$$

where *X*_*B*_ is the current global optimal location. *β* is a normal distribution of random numbers with a mean value of 0 and a variance of 1, called the step size control parameter. *u* ∈ [−1,1] is a random number, which controls the direction of the sparrow movement as well as the step. *f*_*r*_ is the fitness value of the present sparrow, *f*_*B*_ and *f*_*W*_ are the current global best and worst fitness values, respectively. *ε* is the smallest constant to avoid zero-division-error. When *f*_*r*_=*f*_*B*_, this means that the sparrow individuals in the middle of the population are aware of the danger of predation and immediately move closer to others to reduce their risk. When *f*_*r*_ > *f*_*B*_, this represents that the current sparrows are located at the edge of the population and highly vulnerable to predation.

### 2.6. The Proposed SSA-PNN Model

The classiﬁcation performance of PNN model is significantly affected by the smoothing factor *σ*. If the value of smoothing factor is too large, the network model is to convert into a linear classifier, which cannot achieve a fine discrimination for different types with less distinct boundaries. If the value of the smoothing factor is too small, it is equivalent to a nearest neighbor classifier, which only isolates the training samples. The selection of smoothing factor in traditional PNN often depends on manual experience, which cannot get the optimal smoothing factor. To improve the classiﬁcation performance of the PNN network, the SSA algorithm is used to search for the most suitable smoothing factor to construct a SSA-PNN fault diagnosis model. The process of SSA-PNN model is as follows: inputting the training sample data, setting the initial position, population size, and maximum number of iterations, and calculating the fitness value (i.e. the relative error between the predicted value by PNN and the actual value) of the individual position (i.e. the smoothing factor in PNN). Comparing the fitness value obtained for the current and the previous iteration, if the fitness value is better than the previous iteration, the optimal fitness value and its corresponding position are retained.

Repeat the above process until the iteration termination condition is satisfied and the optimal smoothing factor of the PNN can be obtained to construct the SSA-PNN model. The optimization process of the SSA-PNN application steps are as follows:

  Step 1. Select the processed data as the training sample, and take different fault classes as different labels to build the dataset.
  Step 2. Initialize SSA-related parameters, including the number of population, upper and lower boundaries, maximum number of iterations, the proportions of discoverers and scouters in the total population, the early warning value, and set the initial smoothing factor of the PNN network.
  Step 3. Take the error recognition rate of training samples by PNN classification as the fitness function, calculate and sort the initial fitness value to obtain the global worst and best fitness value.
  Step 4. Update the locations of the discoverer, follower, and scouter according to formulas (13)–(15).
  Step 5. Obtain the current fitness value based on the new updated location and compare it with the previous optimal value. If the new location is better than before, update it.
  Step 6. Repeat steps 3 to 5 within the maximum number of iterations, and continuously adjust the smoothing factor to maximize the accuracy of classification during the optimization process.
  Step 7. Output the global optimal value and optimal ﬁtness value, and build the SSA-PNN model by the obtained optimal smoothing factor.

## 3. Fault Diagnosis Process of the Proposed CEEMD-EE-SSA-PNN Model

Based on the above research, a novel fault diagnosis method for rolling bearings by integrating CEEMD, EE, and PNN optimized by SSA is proposed. The ﬂow chart of the proposed fault diagnosis method is presented in Figure 2, and the specific description of the corresponding steps is given as follows:

  Step 1. Collect the vibration signals of rolling bearings under different operating conditions by acceleration sensors.
  Step 2. Use CEEMD to decompose the original vibration signal of each state to obtain *K* IMF components.
  Step 3. Extract the EE values of the *h* effective IMFs with the relatively large correlation coefﬁcient to form a feature vector, which is divided into a training sample set and a testing sample set.
  Step 4. Initialize the parameters of PNN classiﬁcation, and input the training samples set into the PNN classiﬁcation for training.
  Step 5. Set the initial parameters of SSA, and use the SSA algorithm to optimize the smoothing factor *σ* of PNN.
  Step 6. Substitute the optimized smoothing factor *σ* into PNN for training to establish the SSA-PNN diagnosis model.
  Step 7. Input the testing samples set into the trained SSA-PNN prediction model for fault pattern recognition.

## 4. Simulation Experiment

To illustrate the superiority of CEEMD over EMD and EEMD, a simulation experiment is designed. In this experiment, the simulated signal *x*_s_(*t*) is composed of an intermittent signal *x*_1_(*t*) and three sinusoidal signals with diﬀerent initial phases, amplitudes, and frequencies *x*_2_(*t*), *x*_3_(*t*), *x*_4_(*t*), and the decomposition performance of the three methods in dealing with mode mixing and signal reconstruction are compared and analyzed. The simulated signal is constructed as follows:

(16) $$\begin{array}{c} \left\{\begin{array}{c} x_{1}\left(t\right)=\sin\left(2\pi \times f_{1}\times t\right)\left[e^{-2000{\left(t-0.2\right)}^{2}}+e^{-2000{\left(t-0.5\right)}^{2}}+e^{-2000{\left(t-0.8\right)}^{2}}\right],\\ x_{2}\left(t\right)=\sin\left(2\pi \times f_{2}\times t+\frac{\pi }{2}\right),\\ x_{3}\left(t\right)=2\sin\left(2\pi \times f_{3}\times t+\frac{\pi }{3}\right),\\ x_{4}\left(t\right)=3\sin\left(2\pi \times f_{4}\times t-\frac{\pi }{4}\right),\\ x_{s}\left(t\right)=x_{1}\left(t\right)+x_{2}\left(t\right)+x_{3}\left(t\right)+x_{4}\left(t\right), \end{array}\right. \end{array}$$

where *f*_1_ = 150, *f*_2_ = 75, *f*_3_ = 30, *f*_4_ = 10, the sampling frequency is 1000 Hz, and the sampling time is 1 s. The time domain diagram of the simulated signal is shown in Figure 3.

The decomposed IMFs of the simulated signal by EMD are shown in Figure 4. As can be seen from Figure 4, the waveform of IMF 1 component is influenced by the intermittent signal, which contains not only the intermittent signal *x*_1_(*t*) but also another sinusoidal signal *x*_2_(*t*) with higher frequency. Furthermore, IMF 2 affected by IMF 1 also includes an intermittent signal *x*_1_(*t*) and two low-frequency sinusoidal signals *x*_2_(*t*) and *x*_3_(*t*), which leads to a significant mode mixing in all IMFs and makes it difficult to identify the real physical meaning of each IMF.

The EEMD method was utilized to decompose the same simulated signal, and the decomposed results are shown in Figure 5, in which 500 ensemble members were adopted and the RMS amplitude of the added Gaussian white noise was 0.1 times of the standard deviation of the simulated signal. As shown in Figure 5, the phenomenon of modal mixing of IMF components was greatly suppressed by EEMD, the intermittent signal *x*_1_(*t*) was concentrated with the added white noise in IMF 1, IMF 2 approximately agreed with sinusoidal signal *x*_2_(*t*) in the original simulation signal, IMF 3 and IMF 4 corresponded to sinusoidal signal *x*_3_(*t*) and *x*_4_(*t*) in the simulation signal, respectively, which demonstrated EEMD can effectively solve the problem of mode mixing.

Figure 6 presents the IMFs decomposed from the simulated signal by CEEMD, where the number of total aggregation times was 200 and the RMS amplitude of added white noise was 0.1 times of the standard deviation of the simulated signal. The decomposition results are similar to those obtained by EEMD. As can be seen from Figure 6, IMF 1 has a little of a mixture of the intermittent signal *x*_1_(*t*) contaminated to a certain extent by the added noise, and the sinusoidal waveforms *x*_2_(*t*), *x*_3_(*t*), and *x*_4_(*t*) as the components of the original simulated signal were well reconstructed in the corresponding IMFs.

However, in fact, there is a significant difference between the signal reconstructed through IMFs and the original signal. To evaluate the decomposition performance, the reconstruction error (RE) is defined as the difference between the reconstructed and the original signal and is shown in Figure 7. As can be seen from Figures 7(a) and 7(b), the reconstruction error derived from EEMD and CEEMD is very different, the average amplitude of the former is around 0.05, while the corresponding value of the latter is only 10^−15^. The results of simulation experiments indicate that CEEMD not only solves the mode mixing problem of EMD but also overcomes the drawback of incompleteness in signal reconstruction with added white noise in EEMD.

## 5. Experimental Research

### 5.1. Experimental Data

To validate the performance of the proposed method for fault diagnosis of rolling bearings, the experimental dataset is from the bearing database of Case Western Reserve University (CWRU) [46]. The bearing experimental device mainly includes motor, torque sensor, power tester, and electronic control equipment.

The speed of the motor was 1797 r/min and the sampling frequency of the vibration signal was set to 12 kHz, the load was 2 hp, and the sampling time was 10 s. The vibration signals of the SKF6025 bearing were collected by accelerated transducers at the driving end with two different fault diameters of 7 mil and 14 mil (1 mil = 0.001 inches), respectively. There are three kinds of bearing faults generated by electro-discharge machining, including inner ring fault, outer ring fault, and roller fault. In this study, the vibration datasets under six operating conditions were collected, including one normal bearing and five fault bearings. To facilitate classification, the six fault types with different fault locations and fault sizes are artiﬁcially set as class labels 1 to 6: Nor, I07, O07, R07, I14, and O14. The collected vibration signals in each state were divided into 50 groups of samples, each of which contained 2400 sampling points. These fault samples were divided into 30 training samples for training the network and 20 testing samples for verifying the effectiveness of the fault diagnosis model, respectively. The detailed description of the analysis samples in different states and the parameters of the bearing are shown in Table 1. Take one sample of the original vibration signal for each fault type, and the time domain waveforms of ﬁrst 0.2 s in six working conditions of rolling bearings are shown in Figure 8.

### 5.2. Signal Decomposition by CEEMD

Comparing the time domain waveforms of vibration signals in different states of the bearing in Figure 8, it can be seen that when the bearing operates in the normal state, the amplitude of the vibration signal is relatively small and the signal is relatively stable; when the bearing is in the fault state, the vibration signal becomes strong and the amplitude of vibration will be increased; when the inner ring or outer ring of the bearing fails, the periodic impact signals will be generated, and the impact of outer ring fault is stronger than that of the inner ring fault; when the roller fails, it generally shows continuous vibration without obvious periodic impact signal. However, it is difficult to directly determine the working state of the bearing according to the vibration signal.

The CEEMD method was adopted to decompose the vibration signals to obtain a series of IMF components with frequencies ranging from high to low, in which the ratio of the RMS amplitude of the added Gaussian white noise to the standard deviation of the vibration signal was 0.1 and the number of aggregation times was set to 200. Then, calculate the correlation coefficients between each IMF component and the original vibration signal.

Figure 9 shows the correlation coefficients of each IMF component with the original signal of the above six bearing states decomposed by CEEMD. As can be seen from Figure 9, almost all correlation coefficients have a significant decrease starting from the 6th IMF, which illustrates that the first five IMF components have a strong correlation with the original signal and can contain the main characteristic information in the original signal. Therefore, the first five IMFs decomposed by CEEMD are selected as the effective components for feature extraction. The first five IMF components of the six fault signals from high frequency to low frequency after CEEMD decomposition are shown in Figure 10.

### 5.3. Feature Extraction by Energy Entropy

The EE value can reflect the uncertainty of the signal distribution in this frequency band, and different EE value distributions can represent the signals of different states of bearing. To verify that the EE value of IMF component can be used as a feature vector of bearing fault, the difference and repeatability of the EE value of IMF components under different operating states of bearing are analyzed, respectively.

The EE values can be calculated for the first five IMF components selected by the correlation coefficient criterion; taking the 1st group sample signal as an example, the distribution of the EE values in six different bearing states is shown in Figure 11. As can be seen from Figure 11, the EE value of each IMF component varies greatly when the bearing works under different states. Among them, the EE value of all IMF components of the bearing in normal state is much greater than that in other fault states. Meanwhile, compared with other fault states, the EE value distribution of each IMF component in normal state is relatively stable. The reason is the fact that there is the greater randomness of the vibration signal in the normal state. When the bearing fails in operation, a resonance will be produced in some frequencies, that is, the EE value of a certain IMF component after the decomposition of the vibration signal under the fault state is much larger than that of other IMF components. As shown in Figure 11, there is always a phenomenon that the amplitude of a certain bar of the same color (i.e., the same fault state) is much greater than that of other bars of the same color. Therefore, the difference of EE value of IMF components can well reflect the characteristics of the bearing under different operating states and can serve as a feature vector of the bearing state.

To verify the repeatability of the EE value of IMF components under the same operating state of the bearing, Figure 12 presents the EE value distribution of different IMF components obtained from 20 groups of vibration data of the bearing under the same fault state. Figures 12(a)–12(f) show the EE values distribution of the first five IMF components under the fault states of Nor, I07, O07, R07, I14, and O14, respectively. It can be seen from Figure 12 that, for the same fault type of bearing, the EE value of the same IMF component has relatively little fluctuation in the 20 groups of samples, and the EE value of each IMF component has good repeatability.

Thus, it can be concluded that the EE value of the IMF component has good difference and repeatability, which can well reflect the different operating characteristics in different states, and can maintain relatively consistent characteristics under the same working state. Therefore, it is reasonable and effective to select the EE value of IMF component as a feature vector for bearing fault diagnosis.

Each of the six vibration signals corresponding to different fault conditions is divided into 50 groups of samples with 2400 sampling points. The energy entropies of IMF components are extracted from each signal sample to reveal the vibration characteristics of the bearing in different working conditions, which are, respectively, plotted in Figure 13. From Figures 13(a)to 13(e), the energy entropies of IMF components of the 50 groups of vibration signal samples under six different operating conditions are, respectively, revealed, which has roughly certain classifiable characteristics but is more or less irregular. For example, the EE value of the 50 groups of vibration signal samples under O14 state were changed unsteadily and rapidly fluctuated in IMF 3 belonging to Figure 13(c). The EE values of the 50 groups of vibration signal samples under the four states (I07, O07, R07, and I14) are nearly close to the same in IMF 4 and IMF 5 as shown in Figures 13(d) and 13(e). In addition, the EE values of the same IMF under different bearing states are a bit of overlap, according to which it is difficult to distinguish the different conditions of the roller bearings. Therefore, it is necessary to adopt an intelligent classiﬁer to improve the accuracy of bearing fault diagnosis.

### 5.4. Fault Diagnosis by SSA-PNN

After completing the feature extraction of the EE values of the IMF component of the vibration signal of a bearing in different states, the EE values need to be converted into the corresponding fault type of bearing state. However, it is hard to form a direct correspondence between the fault types and features of vibration signal of bearings.

To further verify the superiority of the CEEMD in signal processing and the EE value in feature extraction, the feature vector extracted from the EE value by CEEMD decomposition was inputted into the SVM classiﬁer for classiﬁcation firstly, considering SVM is a classical machine learning method with good ability for small sample data processing and classiﬁcation. The SVM classification results of the testing samples are shown in Figure 14, in which the radial basis function is adopted for the kernel function of SVM. As can be seen from Figure 14, there were prediction errors in the fault states of I07, O07, R07, and I14, especially in the R07 state. The total prediction and classification accuracy rate is 89.17%. It can be seen that the CEEMD-EE-SVM model can achieve a relatively good diagnosis result, which can verify the accuracy of the expression of vibration characteristics using the feature vector extracted by the energy entropy.

To improve the accuracy of bearing fault diagnosis and classification, the PNN model is used as the classifier of fault state for rolling bearing pattern recognition in this paper. PNN model based on Bayesian strategy has strong nonlinear classification ability and does not require backpropagation optimization parameters and training weights. The default value of the smoothing factor in the traditional PNN model is 1.0. During the actual calculation, the smoothing factor was selected manually by continuously examining the classification performance. When the value of the smoothing factor is 0.15, the network classification effect is optimal, that is, the value of smoothing factor in the traditional PNN model is set to 0.15. For the 50 groups of data samples, 30 groups of samples were randomly selected as the training samples and the other 20 groups of samples were used as the testing samples.  Figure 15 shows the training results of the traditional PNN. As can be seen from Figure 15, the training accuracy rate of the CEEMD-EE-PNN model is 96.67%. To further test the classification performance of the PNN, the remaining 20 groups of testing samples were classified and predicted through the PNN model trained by the above 30 groups of samples. The classification result is shown in Figure 16. It can be seen from Figure 16 that several groups of testing samples have made wrong predictions, and the prediction accuracy rate of the CEEMD-EE-PNN model for testing samples is 90.83%, which indicates that the PNN can be applied to the fault diagnosis of rolling bearings.

In this paper, the proposed CEEMD-EE-SSA-PNN model of fault diagnosis with powerful nonlinear approximation and self-learning ability is constructed to complete the classification process from feature vectors to fault type. To obtain higher-precision fault classification results, the SSA algorithm is used to optimize the smoothing factor in the PNN network.

The initial parameters of SSA algorithm were set: the population size of sparrows was 20, the maximum number of iterations was 30, the initial positions of sparrows were randomly generated, the proportions of discoverers and scouters accounted for 70% and 20% of the total population, respectively, the safety threshold was 0.6, and the smoothing factor was the positions of individual sparrow. The relative error of the predicted value and the actual value of 40 training samples trained by the PNN model is used as the fitness function to find the optimal smoothing factor. When the relative error is the smallest, the classiﬁcation result of training samples has the highest accuracy, that is, the fitness value is optimal. The positions of individual sparrows at this time can be obtained as the optimal parameter to the smoothing factor in PNN for constructing the SSA-PNN model.

To verify the superiority of SSA algorithm in optimizing the smoothing factor of PNN, a performance comparison among several optimization methods is conducted, including SSA, PSO, and GA.  Figure 17 shows the change curve of the ﬁtness of different algorithms in the optimization process for PNN, which can well show the optimization process of various algorithms for comparison. As can be seen in Figure 17, the SSA algorithm reaches a local optimal value for the first time at the 2nd iteration and then jumps out of the local optimum at the 5th iteration to continue the optimization search. Finally, SSA achieves the global optimum with the fitness value of 0 at the 8th iteration, which indicates the relative error between the output value of the training sample and the actual value is 0. When the position of individual sparrows at this time is 0.0067, the recognition accuracy rate of the PNN model can reach 100%. Therefore, the best smoothing factor of the PNN model is selected to be 0.0067 by using SSA, which can be used to construct a new trained SSA-PNN model. In contrast, the other two optimization algorithms take several iterations to struggle to escape the local optimum. The fitness begins to decline at the 4th and the 5th iteration in PSO and GA, respectively. PSO algorithm has relative quick convergence ability and converges continuously until the 19th iteration to the minimum. And, GA reaches the local maximum at the 5th iteration and escapes to achieve the minimum at the 18th iteration. It can be seen that compared with PSO and GA, SSA has strong global search ability and can quickly escape the local optimum to achieve the global optimum.

To compare the performance of training results between CEEMD-EE-PNN and CEEMD-EE-SSA-PNN, the same experimental datasets are used to identify the operating state of rolling bearings. The classiﬁcation results of training samples of SSA-PNN are shown in Figure 18. It can be seen from Figure 18, after training on PNN by using the SSA algorithm, the predicted value is consistent with the actual value and the training accuracy rate is 100%.  Figure 19 shows the prediction results of the 20 groups of testing samples by the CEEMD-EE-SSA-PNN network. As can be seen from Figure 19, the classification accuracy rate of the rolling bearing fault state predicted by the CEEMD-EE-SSA-PNN model is 99.17%, which indicates that the improvement of the CEEMD-EE-PNN model optimized by SSA algorithm is eﬀective and can improve the recognition accuracy of rolling bearings fault diagnosis. The SSA algorithm has strong global optimization ability to solve the problem of falling into a local optimum. As can be seen from Figure 19, only one identification error occurs in the status of class label No. 5 (corresponding to fault state I14) for the testing samples set, and its status is mistaken for that of class label No. 4 (corresponding to fault state R07). The main reason lies in the information extraction with the EE value as a single feature vector in the proposed method. For feature extraction, the desired feature vectors have the property that the features of samples belonging to the same states are very similar, while the features of samples belonging to different states are quite different, and that the features are insensitive to information outside the states. It can be seen from the analysis of feature extraction by energy entropy in the previous Section 5.3 that the EE value can well reflect the different states with good difference and repeatability as a feature vector, and meanwhile, it greatly reduces the number of data dimensions that the PNN model needs to process. But the EE values of all IMFs under fault state I14 (corresponding to class label No. 5) are almost indistinguishable from the other states, as shown in Figures 13(a)–13(e). Furthermore, the EE values of I14 state and R07 state overlap very highly in IMF 1, IMF 2, and IMF 3 from Figures 13(a)–13(c), although those of the other states are relatively good, which may cause identification confusion between fault state I14 and fault state R07, and result in the classification of fault state I14 with relatively low accuracy in the actual fault diagnosis. Fortunately, the PNN model optimized by SSA effectively improves the identification accuracy in fault diagnosis of rolling bearings. In addition, the classiﬁcation performance of CEEMD-EE-PNN model on the testing samples set does not reach the accuracy of the training samples set, which indicated that there may be some over-fitting problems in the training process of PNN.

The comparison of the fault diagnosis accuracy of testing samples by using the PSO-PNN, GA-PNN, and SSA-PNN combined with the same signal processing and feature extraction method is shown in Table 2. It can be seen from Table 2 that the proposed CEEMD--EE-SSA-PNN model has the highest accuracy of 99.17% in the fault diagnosis of rolling bearings, the average classification accuracy rate of CEEMD--EE-PSO-PNN is 95.83%, and the CEEMD--EE-GA-PNN gets 93.33% accuracy. These results show that SSA-PNN is superior to the other two PNN models optimized by PSO and GA in fault diagnosis of rolling bearings, indicating that the SSA algorithm can effectively overcome the problem of parameter selection of the PNN model.

The classification results of CEEMD-EE-SVM and CEEMD-EE-PNN are shown in Table 2. As can be seen from Table 2, the CEEMD-EE-SVM and CEEMD-EE-PNN methods have many recognition errors in the fault diagnosis of rolling bearings, and their accuracy rate is lower than that of the CEEMD-EE-SSA-PNN method, which reaches 89.17% and 90.83%, respectively. While in the CEEMD-EE-SSA-PNN model, only one group of diagnostic errors exists in the I14 state, and the different fault states have achieved accurate classification with a prediction accuracy rate of 99.17%. Compared with the two other classifiers, the recognition accuracy of the CEEMD-EE-SSA-PNN model is signiﬁcantly higher for testing samples. These results show that CEEMD-EE-SSA-PNN is superior to the other two classifiers in fault diagnosis of rolling bearings.

To further verify the classification performance of different signal processing methods such as EMD and EEMD when using the same SSA-PNN classifier model, the comparative tests of the EMD-EE-SSA-PNN and EEMD-EE-SSA-PNN methods were carried out. After using the EMD and EEMD methods to decompose the original vibration signal under six different operating states to obtain the effective IMF components, the EE values were extracted to form a feature vector and divided into 30 groups of training samples and 20 groups of testing samples. The classiﬁcation results of EMD-EE-SSA-PNN and EEMD-EE-SSA-PNN models for different fault types are shown in Table 2. It can be seen from Table 2 that EMD-EE-SSA-PNN and EEMD-EE-SSA-PNN have much errors in the fault diagnosis of rolling bearings with the prediction accuracy rate of 88.33% and 91.67%, respectively, and their accuracy is lower than that of the proposed CEEMD-EE-SSA-PNN method. From Table 2, it is obvious that the fault diagnosis rate by using CEEMD is superior to the other two signal processing methods, which further proves that CEEDM has excellent decomposition performance for vibration signal of rolling bearings.

These results all reﬂect that the CEEMD-EE-SSA-PNN method is superior to other methods with higher diagnostic accuracy and is suitable as a powerful model tool for rolling bearing fault diagnosis.

## 6. Conclusions

In this paper, a novel fault classiﬁcation model for rolling bearings is proposed with a combination of CEEMD, EE, and SSA-optimized PNN to identify different fault states of rolling bearings accurately and efﬁciently. Experimental analysis shows that the method has excellent diagnostic performance in rolling bearing fault diagnosis. In the proposed method, the vibration signal is firstly decomposed by CEEMD into a set of IMF components, and the correlation coefficient is used as a selection criterion to determine the effective IMF components to remove noise interference and retain signal features. Compared with EMD, EEMD, and VMD, CEEMD can effectively suppress the adverse effects of noise on signal features, solve the problem of mode mixing in signal decomposition, and overcome the difﬁculty of parameter selection in VMD, which is beneficial to improve the performance of fault diagnosis. Then, the EE value can be used to extract the features of rolling bearing vibration signal for the identification of different fault states with its good difference and repeatability, and the feature set can be input into the classiﬁer to realize the automatic diagnosis of different faults. It is proved that the extraction method of fault feature based on EE can suppress the influence of the redundant information of the fault features, which is useful for improving the classification efficiency. Finally, SSA was introduced to optimize the smoothing factor, which is an important parameter of PNN, to reduce the influence of human factors on the neural network and improve the performance of the fault diagnosis model. Compared with other optimization algorithms, SSA can enhance the global converge ability of the PNN model to prevent falling into the local optimum. The effectiveness and superiority of the proposed method is veriﬁed by using the fault diagnosis of six vibration signals collected from the CWRU bearing dataset. The experimental results demonstrated that the proposed CEEMD-EE-SSA-PNN method has outperformed other methods with better fault diagnosis performance for rolling bearings, and the identiﬁcation accuracy rate reaches 99.17%.

In the future, we will study advanced feature extraction methods based on multi-sensor information fusion to further improve the pattern identiﬁcation results. Meanwhile, we will investigate the latest deep learning algorithms applied to bearing failure diagnosis to improve the efficiency and precision of the classification model. In addition, development of online intelligent bearing fault diagnosis technology to realize real-time condition monitoring and fault diagnosis of rolling bearings is also worth further study.

## Figures and Tables

**Figure 1:** Probabilistic neural network structure diagram.

**Figure 2:** Flow chart of the proposed CEEMD-EE-SSA-PNN model for fault diagnosis.

**Figure 3:** Time domain diagram of the simulated signal.

**Figure 4:** Decomposed IMFs of the simulated signal by EMD.

**Figure 5:** Decomposed IMFs of the simulated signal by EEMD.

**Figure 6:** Decomposed IMFs of the simulated signal by CEEMD.

**Figure 7:** Reconstruction error derived by EEMD and CEEMD. (a) EEMD. (b) CEEMD.

**Figure 8:** Time domain diagram of rolling bearings under six working conditions.

**Figure 9:** Correlation coefficients between each IMF component and the original signal.

**Figure 10:** CEEMD decomposition results of different states. (a) Nor. (b) I07. (c) O07. (d) R07. (e) I14. (f) O14.

**Figure 11:** Difference of energy entropy of IMF components in different states.

**Figure 12:** Repeatability of energy entropy of IMF components in different fault states. (a) Nor. (b) I07. (c) O07. (d) R07. (e) I14. (f) O14.

**Figure 13:** Energy entropy distribution of IMFs in different fault states. (a) IMF 1. (b) IMF 2. (c) IMF 3. (d) IMF 4. (e) IMF 5.

**Figure 14:** Classiﬁcation results of CEEMD-EE-SVM.

**Figure 15:** Classiﬁcation results of training samples of CEEMD-EE-PNN.

**Figure 16:** Classiﬁcation results of testing samples of CEEMD-EE-PNN.

**Figure 17:** Fitness value curve of different optimization methods.

**Figure 18:** Classiﬁcation results of training samples of CEEMD-EE-SSA-PNN.

**Figure 19:** Classiﬁcation results of testing samples of CEEMD-EE-SSA-PNN.

**Table 1:** Description of the experimental dataset.

Label	Fault type description	Abbreviation of fault type	Fault size (mil)	Training sample number	Testing sample number
1	Normal	Nor	0	30	20
2	Inner ring fault	I07	7	30	20
3	Outer ring fault	O07	7	30	20
4	Roller fault	R07	7	30	20
5	Inner ring fault	I14	14	30	20
6	Outer ring fault	O14	14	30	20

**Table 2:** Accuracy comparison of different methods.

Methods	Fault type (group)						Accuracy (%)
	Nor	I07	O07	R07	I14	O14	
CEEMD-EE-SVM	20/20	19/20	19/20	11/20	18/20	20/20	89.17 (107/120)
CEEMD-EE-PNN	20/20	20/20	20/20	13/20	17/20	19/20	90.83 (109/120)
EMD-EE-SSA-PNN	20/20	18/20	18/20	13/20	17/20	20/20	88.33 (106/120)
EEMD-EE-SSA-PNN	20/20	19/20	19/20	15/20	18/20	19/20	91.67 (110/120)
CEEMD-EE-PSO-PNN	20/20	20/20	20/20	17/20	18/20	20/20	95.83 (115/120)
CEEMD-EE-GA-PNN	20/20	20/20	20/20	15/20	18/20	19/20	93.33 (112/120)
CEEMD-EE-SSA-PNN	20/20	20/20	20/20	20/20	19/20	20/20	99.17 (119/120)

## Data Availability

The data used to support the ﬁndings of this study are available from the corresponding author upon request.
